The article "Effect of the new synthetic vitamin E derivative ETS-GS on radiation enterocolitis symptoms in a rat model" was published in 2013. Journal: Oncol Lett.

# Effect of the new synthetic vitamin E derivative ETS-GS on radiation enterocolitis symptoms in a rat model

**DOI:** 10.3892/ol.2013.1581

**Published:** 2013-09-12

**Authors:** SATOSHI SUGITA, MASAFUMI INOMATA, YOHEI KONO, HIDEFUMI SHIROSHITA, TSUYOSHI ETOH, NORIO SHIRAISHI, SEIGO KITANO

**Affiliations:** Department of Gastroenterological and Pediatric Surgery, Oita University Faculty of Medicine, Yufu, Oita 879-5593, Japan

**Keywords:** radiation enterocolitis, vitamin E derivative, apoptosis

## Abstract

Radiation enterocolitis is a severe adverse event that occurs after radiotherapy for malignant abdominal tumors. In this study, the therapeutic effects of ETS-GS, a novel vitamin E derivative with antioxidative and anti-inflammatory abilities, were examined in a rat model of radiation enterocolitis. The radiation enterocolitis model was created by irradiation of male rats with a single dose of 10 Gy. ETS-GS was administered subcutaneously (10 mg/kg/day) for five consecutive days from two days prior to irradiation. The animals were sacrificed three days after irradiation; following which, ileal tissue samples were analyzed for macroscopic and histological findings, presence of apoptosis, degree of oxidative stress and inflammation. In the irradiated group, severe erosion was observed in the small intestine in addition to necrosis of the mucosal layer, swelling and invasion of inflammatory cells of the submucosal layer, and shortening of the crypts. In irradiated rats that received ETS-GS, mucosal injury in the small intestine was milder compared with that of irradiated rats that received no ETS-GS. In addition, ETS-GS decreased apoptosis in the small intestine and reduced the activity of myeloperoxidase and malondialdehyde, which are markers for inflammation and oxidative stress. ETS-GS with antioxidant activity has a therapeutic effect on the symptoms of radiation enterocolitis in a rat model.

## Introduction

Radiation enterocolitis is a severe adverse event resulting from radiation therapy for abdominal and pelvic malignancies (1,2). As administration of radiation therapy has increased in recent years, the incidence of radiation enterocolitis has also increased (3). Drug therapies for the treatment of radiation enterocolitis include antispasmodic, antidiarrheal, steroidal (4,5) and nonsteroidal anti-inflammatory agents, such as sulfasalazine (4) and aspirin (6,7). In cases refractory to treatment using these drugs, surgical treatment is often considered. Therefore, the development of new and more effective drugs for the treatment of radiation enterocolitis is desirable.

Certain studies have suggested that radiation enterocolitis is caused by oxidative stress, as antioxidants including aminoguanidine, octreotide and glutamine have been shown to improve radiation enterocolitis in animal models (8–10). In this study, a new antioxidant agent, ETS-GS (γ-L-glutamyl-S-[2-[[[3,4-dihydro-2,5,7,8-tetramethyl-2-(4,8,12-trimethyltri-decyl)-2H-1-benzopyran-6-yl]oxy]carbonyl]-3-oxo-3-[(2-sulfoethyl)amino]propyl]-L-cysteinylglycine sodium salt), was developed for the treatment of radiation enterocolitis. This agent is soluble and stable in water, and has high antioxidative and anti-inflammatory activity. Several studies have validated the antioxidative and anti-inflammatory effects of this agent (11–15).

The article "Effect of the new synthetic vitamin E derivative ETS-GS on radiation enterocolitis symptoms in a rat model" was published in 2013. Journal: Oncol Lett.

In the present study, the therapeutic effects of this new vitamin E derivative, ETS-GS, were examined in a rat model of radiation-induced enterocolitis.

## Materials and methods

### Chemicals

The vitamin E derivative ETS-GS consists of chemically linked vitamin E, glutathione, taurine and malefic acid. The sterile, aqueous solution of ETS-GS used in this experiment was provided by Oga Research Inc. (Osaka, Japan; Fig. 1).

### Animals

Six-week-old male Sprague-Dawley rats (Kyudo, Saga, Japan) weighing 150–250 g (n=27) were used in all experiments. The rats were housed in cages controlled for temperature (22±2°C), humidity and lighting (12-h light/dark cycle), with free access to water and food. The study protocol was approved by the Animal Ethics Committee of Oita University Faculty of Medicine (Yufu, Japan).

### Experimental protocol

Rats were randomly divided into three groups (n=9 per group) according to treatment. The untreated group received no radiation and no treatment, the irradiated (IR) group received abdominal radiation, and the IR + ETS-GS group received abdominal radiation and ETS-GS treatment. ETS-GS (10 mg/kg dissolved in 0.9% NaCl) was administered subcutaneously for five consecutive days commencing two days prior to radiation exposure. The dose of ETS-GS was determined according to the protocol in a previous study using this rat model (12–14).

Prior to irradiation, rats were anesthetized by intraperitoneal injection of sodium pentobarbital (Nembutal; Dainippon Sumitomo Parma Co., Ltd., Japan) at a dose of 50 mg/kg body weight, and placed in the supine position. They were then irradiated with a single dose of 10 Gy to the whole abdomen using a Gammacell 40 Extractor (Atomic Energy of Canada Ltd., Chalk River, ON, Canada). Modified lead plates were used to shield the head and chest of the rats during irradiation. Three days after irradiation, rats were sacrificed humanely according to the Institutional Animal Care and Use Committee guidelines of Oita University. The terminal ilea were harvested for analysis, and a portion was fixed in buffered formalin for histopathological examination. The remainder tissue was stored at −80°C for biochemical analysis.

The article "Effect of the new synthetic vitamin E derivative ETS-GS on radiation enterocolitis symptoms in a rat model" was published in 2013. Journal: Oncol Lett.

### Histopathological analysis

After washing with saline solution, ileal tissue specimens were fixed in 10% buffered formaldehyde and embedded in paraffin, and 5*-*μm sections were prepared using a microtome. Sections were stained with hematoxylin and eosin and analyzed for morphological changes.

### Detection of DNA fragmentation

Using the terminal deoxynucleotidyl transferase (dUTP) nick-end labeling (TUNEL) method, DNA fragmentation was detected under a fluorescent microscope, and flow cytometry was performed promptly. Highly sensitive and specifically labeled fluorescein dUTP is labeled on the free 3′-OH end of fragmented DNA of the cell, after which terminal transferase causes apoptosis. Staining was performed using an MK500 *In situ* Apoptosis Detection kit (Takara Bio Inc., Otsu, Japan) according to the manufacturer’s instructions. In total, 1000 cells, including cells positive for TUNEL, were counted in 10 random high-power fields (x400 magnification), and the percentage of TUNEL-positive cells was used to calculate the apoptotic index (16,17).

### Caspase-3/7 activity

Caspases are a group of cysteine proteases that constitute a signaling pathway which causes cells to undergo apoptosis. Caspase-3/7, also known as effector caspases, are activated by initiator caspases. They work to disassemble other intracellular proteins and increase apoptosis; in cells undergoing apoptosis, caspase-3/7 activity is enhanced (18,19). Caspase-3/7 activity was measured in this study using a Caspase-Glo^®^ 3/7 assay kit (Promega Co., Madison, WI, USA) according to the manufacturer’s instructions.

### Biomarker assays

Intestinal myeloperoxidase (MPO) activity was assayed using a rat MPO enzyme-linked immunosorbent assay (ELISA) kit (Hycult^®^ Biotech, Uden, The Netherlands) according to the manufacturer’s instructions. MPO is a peroxidase enzyme most abundant in neutrophil granulocytes (20). Malondialdehyde (MDA) in the ileal tissue was assayed to assess the degree of oxidative stress using a commercial kit for thiobarbituric acid reactive substances (Northwest Life Science Specialties LLC, Vancouver, WA, USA). Absorbance at 532 nm was determined using an ELISA plate reader (Bio-Rad Laboratories, Hercules, CA, USA).

### Statistical analysis

All data are expressed as the mean ± standard deviation. One-way analysis of variance was used for statistical analysis, and P<0.05 was considered to indicate a statistically significant difference. The Dr. SPSS II statistical software (SPSS, Inc., Chicago, IL, USA) was used to evaluate the data.

The article "Effect of the new synthetic vitamin E derivative ETS-GS on radiation enterocolitis symptoms in a rat model" was published in 2013. Journal: Oncol Lett.

## Results

### Macroscopic and histopathological findings

In this study, no treatment-related mortality occurred in any rats. In the IR group, histological examination showed severe erosion, necrosis of the mucosal layer, swelling and invasion of inflammatory cells of the submucosal layer, and shortening of the crypts in the ileum (Fig. 2). In the IR + ETS-GS group, ileal injury was improved compared with that of the IR group. In addition, rats administered only ETS-GS were histologically similar to the untreated group in the preliminary experiment (data not shown).

### Assessment of apoptosis using the TUNEL method and caspase-3/7 activity

TUNEL staining and caspase-3/7 assay were used to evaluate apoptosis in ileal tissue specimens. In the IR group, numerous dyed apoptotic cells were confirmed in the mucosal layer of the intestine. By contrast, very few dyed apoptotic cells were observed in the specimens obtained from the untreated and IR + ETS-GS groups (Fig. 3). The apoptotic index of the IR group was significantly higher than that of the untreated group (186±41.1 vs. 28.3±17.6, P<0.05) (Fig. 4). In the IR + ETS-GS group, the apoptotic index was lower than that in the IR group (27.7±3.5 vs. 186±41.1, P<0.05).

In the IR group, intestinal caspase-3/7 activity was found to be significantly increased compared with that in the untreated group (1.89±0.42 vs. 1.00±0.45, P<0.05); however, ETS-GS significantly decreased this activity (0.71±0.56) (Fig. 5).

### MPO activity

The activity of intestinal MPO was measured to assess the degree of inflammation. Intestinal MPO activity in the IR group was significantly higher than that in the untreated group (1394.0±375.6 vs. 510.3±141.8 ng/ml, P<0.05). In the IR + ETS-GS group, MPO activity was significantly decreased compared with that in the IR group (925.0±196.7 vs. 1394.0±375.6 ng/ml, P<0.05) (Fig. 6).

### MDA assay

The activity of intestinal MDA was measured to assess the degree of oxidative stress. MDA is formed by oxidation of lipids and is an indicator of oxidative stress (21). In the IR group, the intestinal MDA level was found to be significantly increased compared with that in the untreated group (0.07±0.01 vs. 0.04±0.02, P<0.05). Treatment with ETS-GS significantly decreased the MDA level compared with that of the IR group (0.04±0.01 vs. 0.07±0.01, P<0.05) (Fig. 7).

## Discussion

To the best of our knowledge, this is the first study demonstrating the effect of the new vitamin E derivative ETS-GS on radiation enterocolitis in rats. Histopathological analysis showed that administration of ETS-GS decreased the degree of mucosal erosion and necrosis, swelling and invasion of inflammatory cells of the submucosal layer, and shortening of the crypts caused by acute radiation enterocolitis. This biological activity was associated with caspase-3/7 levels, apoptotic index, and MPO and MDA levels in ileal tissue specimens of rats treated by administration of ETS-GS.

The article "Effect of the new synthetic vitamin E derivative ETS-GS on radiation enterocolitis symptoms in a rat model" was published in 2013. Journal: Oncol Lett.

Several animal models of radiation enterocolitis have been developed. Mylonas *et al* prepared a model by abdominal irradiation of a single dose of 11 Gy in rats (22), while Wang *et al* created a model by irradiating once daily 4.2 Gy for 16 days (23). In this study, the radiation enterocolitis model was created by irradiation of a single dose of 10 Gy to male rats. This method was successful in inducing radiation enterocolitis. Examinations were performed with future clinical application in mind. Huang *et al* administered aminoguanidine prior to irradiation when examining the effects of this agent on small bowel damage in rats, to demonstrate its prophylactic effect (8). By contrast, Emami *et al* administered aminoguanidine after irradiation, with the intention of showing its therapeutic effect (24). In the present study, the drug was administered prior to and after irradiation, consecutively for five days. As a result, the onset of radiation enterocolitis was significantly suppressed. In addition, a similar effect was observed after administration of ETS-GS (10 mg/kg), with no significant toxicity, as observed in previous studies (12–14).

Abdominal irradiation causes inflammation of the intestinal tract with submucosal edema, hyperemia and infiltration of the lamina propria due to the activation of inflammatory cells (24). Radiation energy absorbed by the body is supplied to biopolymers, such as nucleic acids and proteins, as well as to *in vivo* water molecules. These molecules are then ionized or energized, thereby inducing radiation damage (25,26). Radiation injury can be caused by direct or indirect action (27). Direct action causes damage directly to the biopolymers, and indirect action causes ionization and dissociation of water molecules. With indirect action, free radicals and reactive oxygen species are formed through secondary chain reactions, inducing apoptosis and tissue damage. Furthermore, Hepgül *et al* and Mollà *et al* reported the involvement of oxidative stress in radiation-induced enterocolitis (28,29). MPO exists in abundance in neutrophils and is used as a marker for the detection of neutrophil accumulation within inflamed tissue (20). MDA is formed by oxidization of lipids and is an indicator of oxidative stress (21). Caspase-3/7 is activated by initiator caspases, such as caspase-8/9; these caspases break down proteins within cells and trigger apoptosis, which is why they are used as markers of apoptosis (18,19). In this experiment, dysfunction of the ileal mucous membrane as a result of radiation exposure was inhibited through ETS-GS administration, and ileal MPO, MDA and caspase-3/7 protein activity was significantly decreased. Based on these findings, we suggest that oxidative stress, which occurs due to radiation enterocolitis, is impeded by administration of ETS-GS, and tissue damage is prevented through inhibition of apoptosis.

The article "Effect of the new synthetic vitamin E derivative ETS-GS on radiation enterocolitis symptoms in a rat model" was published in 2013. Journal: Oncol Lett.

ETS-GS is highly soluble in water and has both antioxidant and anti-inflammatory actions, including suppression of MDA, interleukin-6 and tumor necrosis factor-α (13,14). As ETS-GS dissolves easily in water, administration not only by subcutaneous injection but also by intravenous injection and drip infusion may be possible. Intravenous injection of ETS-GS has been shown to improve lipopolysaccharide-induced acute lung and liver injury and renal ischemia reperfusion in rat models, with no reports of apparent side-effects (13,14). Numerous reported therapeutic agents for the treatment of radiation enteritis must be administered orally (30–32). ETS-GS has the advantage that it may be administered intravenously to patients with radiation-induced enterocolitis for whom oral administration is not possible.

The present study is an animal experiment using rat models; however, the results for clinical application were encouraging. For clinical purposes, the mechanism of the agent must be clarified in more detail, and the presence or absence of side-effects must be confirmed. Radiation is utilized in the treatment of malignant tumors; the effects of ETS-GS administration on these tumors and its interaction with radiation therapy also require clarification. A previous study demonstrated the antiproliferative effects of a new α-lipoic acid derivative, DHL-HisZnNa, with strong antioxidant action similar to that of ETS-GS, in HT29 human colon cancer cells *in vitro*(33). Similar effects are predicted for ETS-GS, and future studies must verify this hypothesis.

In conclusion, this study demonstrated that a new synthetic vitamin E derivative, ETS-GS, has therapeutic effects against the intestinal damage caused by abdominal irradiation, through reduction of the inflammatory response, apoptosis and oxidative stress.

## Figures and Tables

**Figure 1:** Structure of ETS-GS (γ-L-Glutamyl-S-[2-[[[3,4-dihydro-2,5,7,8-tetramethyl-2-(4,8,12-trimethyl-tri-decyl)-2H-1-benzopyran-6-yl]oxy]carbonyl]-3-oxo-3-[(2-sulfoethyl)amino]propyl]-L-cysteinylglycine sodium salt).

**Figure 2:** Histopathological changes in ileal tissue after irradiation. Ileal tissues were fixed, embedded, sectioned and stained with hematoxylin and eosin. No histological alternations were observed in (A) the untreated group, whereas severe erosion, necrosis of the mucosal layer, swelling and invasion of inflammatory cells of the submucosal layer, and shortening of the crypts were observed in (B) the irradiated (IR) group. Attenuated irradiated changes were observed in (C) the IR + ETS-GS group. Magnification, ×200.

The article "Effect of the new synthetic vitamin E derivative ETS-GS on radiation enterocolitis symptoms in a rat model" was published in 2013. Journal: Oncol Lett.

**Figure 3:** Terminal deoxynucleotidyl transferase nick-end labeling staining of an ileal section. (B) Representative histological section from the irradiated (IR) group, in which numerous dyed apoptotic cells are visible (arrows). By contrast, in (A) the untreated group and (C) the IR + ETS-GS group, almost no apoptotic cells were present. Magnification, ×400.

**Figure 4:** Number of apoptotic cells. Terminal deoxynucleotidyl transferase nick-end labeling (TUNEL)-positive cells were counted over 10 fields selected randomly in the field of view, which included 1000 cells, using an optical microscope (magnification, ×400). Results are expressed as the mean ± standard deviation (n=9 per group, ^*^P<0.05).

**Figure 5:** Effect of ETS-GS on caspase-3/7 levels in the ileal tissue of rats following irradiation. Caspase-3/7 levels in the ileal tissues were measured three days after irradiation. Results are expressed as the mean ± standard deviation (n=9 per group, ^*^P<0.05).

**Figure 6:** Effect of ETS-GS on myeloperoxidase (MPO) levels in the ileal tissue of rats after irradiation. The activity of MPO in the ileal tissues was examined three days after irradiation. Results are expressed as the mean ± standard deviation (n=9 per group, ^*^P<0.05).

**Figure 7:** Effect of ETS-GS on malondialdehyde (MDA) levels in the ileal tissue of rats after irradiation. MDA levels in the ileal tissues were measured three days after irradiation. Results are expressed as the mean ± standard deviation (n=9 per group, ^*^P<0.05).
